The article "Assessment of Saudi Women's Adherence and Experience with Venous Thromboembolism Prophylaxis after Cesarean Section Delivery Using Telemedicine Technology" was retracted in 2023. Reasons: signs of a paper mill; compromised peer review; unreliable results or conclusions.

# Assessment of Saudi Women's Adherence and Experience with Venous Thromboembolism Prophylaxis after Cesarean Section Delivery Using Telemedicine Technology

**DOI:** 10.1155/2022/8440789

**Published:** 2022-03-14

**Authors:** Dalia Ahmed Elmaghraby, Zakiah Khalid Al-Bassri, Zainab Ahmed AlTuraiki, Jinan Adnan Alsaleh, Latifah Saleh Alzuwayyid, Norah Abdulmohsen Albanyan, Abdulaziz Saleh Almulhim

**Affiliations:** Department of Pharmacy Practice, College of Clinical Pharmacy, King Faisal University, Al-Ahsa 31982, Saudi Arabia

## Abstract

**Background:**

Telemedicine technology is widely used especially after the COVID-19 pandemic. It can be used to give medical advice as well as follow up with the patients at home in the outpatient setting. Low molecular weight heparin, such as enoxaparin, decreases the risk of venous thromboembolism after cesarean delivery.

**Objective:**

assessing postcesarean women's adherence and experience to enoxaparin thromboprophylaxis regimens in the outpatient setting via telephone calls.

**Methods:**

prospective cohort study was conducted in the Maternity and Children Hospital (MCH). Postcesarean women were interviewed at the postnatal ward in the MCH. The participants were followed up for 10 days of the delivery to assess their adherence to and experience with enoxaparin thromboprophylaxis. Suboptimal adherence was defined as the missing of one or more doses of enoxaparin.

**Results:**

170 women participated in this study. The majority of them (78.8%) were fully adherent to enoxaparin while 21.2% missed at least one dose. The most-reported causes for suboptimal adherence were perceived lack of necessity (44.4%), forget to take the injection (30.6%), feeling of high load going to the primary care unit to take injection (27.8%), and fear of injection (11.1%).

**Conclusion:**

Telemedicine technology could be used to assess patients' adherence. The study results showed that the majority of participants were fully adherent to postcesarean enoxaparin but more than 20% of the participants were suboptimal adherent. Proper patient education techniques could influence patients' adherence and potentially decrease the risk of DVT in those populations.

## 1. Introduction

Venous thromboembolism (VTE), including deep vein thrombosis (DVT) and pulmonary embolism (PE), is one of the main causes of maternal death during and after pregnancy [1, 2]. The risk of VTE is 5-fold increased during pregnancy and 60-fold increased during the postpartum period compared with nonpregnant women [3]. In addition, a meta-analysis was published in 2016 reported that the VTE incidence after a cesarean section (CS) is quadrupled compared to vaginal delivery [4]. The current national and international practice guidelines recommend a short course of thromboprophylaxis following a CS [5–7]. They recommend 10 days of low molecular weight heparin (LMWH) as postnatal thromboprophylaxis in mothers who had emergency CS and for those who underwent elective CS with additional risk factors. Guidelines agreed on the use of enoxaparin as postnatal thromboprophylaxis [5–7]. Revising the risk factors to develop VET, which was described in different international guidelines, revealed that the majority of the Saudi obstetrical population is considered as high risk [8–10]. Examples of these risk factors are multiple pregnancies, obesity (BMI > 30 Kg/m2), advanced maternal age, and repeated cesarean section [5–7]. LMWH is given subcutaneously which may affect the parturients' adherence after hospital discharge [11, 12]. Therefore, it is important to understand and assess postcesarean women's adherence to LMWH thromboprophylaxis regimens in the outpatient setting. Several studies assessed women's adherence and their experiences with LMWH thromboprophylaxis [13–15]. We used telemedicine technology to assess the patient's adherence and experience with LMWH.

## 2. Materials and Methods

### 2.1. Study Design, Sampling, and Data Collection

This was a prospective cohort study conducted in the Maternity and Children Hospital (MCH) in Al-Ahsa region. MCH is the main tertiary care public maternity hospital in Al-Ahsa with a 450-bed capacity [16]. Concerning the sample size, per our institution statistics, there are around 1000 C-section deliveries per year, with a power of 90%, and an adherence rate of 82% a sample of 138 participants would be needed.[11].

Postcesarean parturients were interviewed at the postnatal ward in the MCH by pharmacy interns (Z. K. A., Z.A. A., L.S. A., J.A.A) who were trained and prepared in patients' interviews and data collection to obtain their verbal informed consent and collect their demographics. Exclusion criteria were as follow: age < 18 years and long-term anticoagulation treatment. The participants were followed up after 10 days of the delivery via a telephone call to assess their adherence to and experience with LMWH thromboprophylaxis. Suboptimal adherence was defined as the missing of one or more doses of LMWH. During the hospitalization of the parturients, it was the responsibility of the nurses to inject the patients with the LMWH, and we assume that the adherence rate was 100%. After parturient's discharge, they can choose to inject the LMWH either by themselves, with the help of a family member, or they can be referred to the nearest primary care center and administered by a health care provider (i.e., daily visits to primary care center). The study participants were recruited over four months (from January 2021 to April 2021). Excel spreadsheet was used as a structured data collection tool.

### 2.2. Questionnaire Description

The study questionnaire consisted of 21 questions. Some questions were adopted from a previous study and modified according to the particular Saudi environment [13]. The questionnaire was confirmed for its face and content validity by experts in the field of pharmacy practice at King Faisal University, who have experience in questionnaire development [17, 18] and adjusted after a pilot study conducted on 10 participants. The questionnaire is composed of three main parts. (1) Participant's demographics of age, education and economic level, and pregnancies and abortion numbers. (2) Presence of risk factors that may increase the risk of having venous thromboembolism. (3) Measuring parturients' adherence to LMWH after discharge from the hospital and what kind of problems they faced during using the LMWH.

### 2.3. Ethics

The study was approved by the Institutional Review Board (IRB) at King Fahad Hospital Hofuf (KFHH RCAN0. 07-37-2021) and the MCH Research Ethics Committee (RS-01238). All participants provided informed verbal consent before data collection.

### 2.4. Statistical Analyses

After data were extracted, it was revised, coded, and fed to statistical software IBM SPSS version 22 (SPSS, Inc. Chicago, IL) [19]. Descriptive analysis based on the frequency and percent distribution was done for all variables including demographic data, obstetric and gynecological history, medical and drug history, compliance to LMWH with parturient experience, and beliefs regarding the drug. Continuous variables were described as means ± standard deviation (SD). Univariate relations were used to assess relations between females' adherence to the prescribed LMWH and their bioclinical data, obstetric, and gynecological data, and their experience with LMWH. A *P* value less than 0.05 was considered statistically significant. Appropriate graphs were also generated by GraphPad Prism® version 9.1.2 for Windows (San Diego, CA, USA) [20].

## 3. Results

### 3.1. Participants Characteristics

Two hundred parturients consented to participate in this study. However, only 170 (85%) responded to the telephone call and completed the questionnaire. The mean age was 32.9 ± 6.3 years. Concerning the level of education, 41.2% had a university degree. Regarding the economic status,71% of participants reported a monthly income of less than 10000 SR. For body mass index (BMI), 42.4% were obese. Smoking of husbands was reported by 40% of the participants. Anemia and hypertension were the frequently observed comorbidities (15.9%) and (11.2%), respectively. (Table 1).

### 3.2. Participants' Adherence with LMWH

Following hospital discharge, 134 (78.8%) parturients were fully adherent to the LMWH course, while 36 (21.2%) were suboptimal adherent (Figure 1).

The reported causes of suboptimal adherence were perceived lack of necessity (44.4%), forget to take the injection (30.6%), feeling of high load going to the primary care unit to take injection (27.8%), and fear of injection (11.1%) While 25% mentioned other causes including doctor advise to stop the medication, no one can help in injection administration, all the doses were taken before discharge, misunderstanding of the number of doses, and one injection was damaged. (Table 2.).

No significant differences were observed in the demographic characteristics between LMWH adherent and suboptimal adherent parturients; these included ages, educational level, monthly income, and comorbidities (Table 3.)

The parturients' gynecological and obstetric data examined did not differ between participants with optimal and suboptimal adherence to LMWH; these included gravidity, number of previous normal deliveries, number of previous CS, and number of children (Table 4).

### 3.3. Participants' Experiences and Views regarding LMWH

Concerning parturients' experiences and views regarding LMWH. One hundred twenty-one participants (71.2%), and 9 (5.3%) were educated about the indication and method of administration by physician and pharmacist, respectively. On the other hand, 23.5% of the study participants denied receiving any education about enoxaparin. (Table 5).

Compliance to LMWH was detected among all participants who previously administered enoxaparin three times compared to 50% of those who administered enoxaparin twice before (*P* = .049). Also, 88.2% of females who inject themselves for having the medication were complaint in comparison to 76.4% of those who had the injection by health care staff (*P* = .001) (Table 5).

∗*P* < 0.05 (significant).

The average doses taken of LMWH among the adherent group was 7.4 compared to 3.9 for nonadherent females with statistical significance (*P* = .001) (Table 6).

## 4. Discussion

Our study showed an adherence rate of 78.8% among parturients' who underwent CS. This is consistent with previously published studies [11, 14, 15, 21]. Considering the risk of VTEs following CS, this rate of adherence is reassuring [10]. Unlike the findings in our study, the study by Rottenstreich and colleagues found that optimal adherence was seen in only 67.2%, patients were interviewed at the end of the VTE prophylaxis course which could minimize the observer bias [13]. Concerning causes of suboptimal adherence to LMWH, perceived lack of necessity, forgetting, difficulty going to the primary care unit, and fear of needles were the most common reasons reported by the study participants. Hordern's and colleagues conducted a prospective study to assess patients' compliance with LMWH postnatal thromboprophylaxis, bruising or wound complications, forgetfulness, fear or dislike of needles, and feeling that the injections were not helping were the most common reasons for suboptimal adherence [14]. Regarding LMWH administration, only Fifty-one (30%) of our study participants reported LMWH self-injection. Rottenstreich and colleagues reported that the explanation of the technical administration of LMWH in the hospital before discharge were independent predictors of adherence following discharge [13]. It is worth noting that (82.9%) reported self–injection; nevertheless, adherence was not statistically different regardless of the method of administration [13]. Similarly, Patel and colleagues reported that the majority of the patients self-injected LMWH, again, emphasizing the importance of patient education and counseling [15]. In our study, only forty (23.5%) of the respondents reported that they did not receive LMWH administration instructions. Several studies found proper patients' education and communication were an important factor to increase patient medication adherence to different dosage forms [22–26]. Contrary to ours, Alzoubi and colleagues found that the majority of study participants who underwent CS have not been educated well about thromboembolism complications due to CS [27]. One study done in Memphis found that when the pharmacist followed up their patient by telephone that led to increased patient adherence to their medication and decreases rehospitalization due to disease complications [28]. After the COVID-19 situation, telemedicine is effectively and widely used for patient counseling in Saudi Arabia and worldwide [29–33]. According to the Saudi FDA, The cost of one injection of enoxaparin 40 mg\0.4 ml prefilled syringe is about 39.65 Saudi Riyal which equals to 10.57 United States Dollars. [34] But the drug cost is not a burden to the patients as all Saudi patients are covered by public insurance [35]. The current practice guidelines recommend a short course of thromboprophylaxis following a CS. The Royal College of Obstetricians and Gynecologists (RCOG) recommends 10 days of low molecular weight heparin (LMWH) as postnatal thromboprophylaxis in mothers who had emergency CS, and for those who underwent elective CS with additional risk factors. Also, The American College of Chest Physicians recommends prophylactic LMWH after cesarean delivery if the patients had additional factors that increase their risk for VTE. Similarly, the Australian guideline of King Edward Memorial Hospital recommended LMWH thromboprophylaxis after cesarean birth in elective cesarean with one or more risk factors or in mothers who underwent Emergency/nonelective CS in labor [5–7]. Several studies stated that obesity increases the risk of DVT in pregnancy and the postpartum period [36–39]. The majority of the study participants were obese (42.4%) and overweight (28.8%). The same results were found in different Saudi epidemiological studies which reported increased obesity rates in pregnant and nonpregnant Saudi females [40–44].

Telemedicine technology and following the patient via phone calls are widely used especially during the COVID-19 pandemic. [45–48]. We used this technology in following up with our participants because it is easier and more convenient for postpartum women. Although the current study is based on a single-center experience, it was conducted at the main public maternity hospital in the region. Our study has some limitations. First, due to the nature of the study, patients were interviewed over the phone at the end of the thromboprophylaxis course, this may increase the risk of recall bias. Second, the response rate was 85% and this could have introduced selection bias which could have distorted the adherence rate [49].

## 5. Conclusions

Telemedicine technology could be used to assess patients' adherence. The study results showed that the majority of participants were fully adherent to postcesarean enoxaparin but more than 20% of the participants were suboptimal adherent. Proper patient education techniques could influence patients' adherence and potentially decrease the risk of DVT in those populations.

## Figures and Tables

**Figure 1:** Postdischarge adherence of participants with LMWH for venous thromboprophylaxis after cesarean delivery.

**Table 1:** Demographic and clinical characteristics of the 170 participants.

	Total	
	No	%
Age in years		
<30	52	30.6%
30–39	90	52.9%
40+	28	16.5%
Educational level		
Below secondary	33	19.4%
Secondary	67	39.4%
University	70	41.2%
Monthly income		
<10000 SR	122	71.8%
>10000 SR	48	28.2%
Body mass index		
Normal weight	49	28.8%
Overweight	49	28.8%
Obese	72	42.4%
Smoking (active or passive smoker)		
Nonsmoker	102	60%
Secondhand smokers	68	40%
Comorbidities		
None	112	65.9%
DM	10	5.9%
HTN	19	11.2%
Anemia	27	15.9%
Hypothyroidism	4	2.4%
Others	10	5.9%
Obstetric and gynecological data		
Gravidity		
1–2	42	24.7%
3–5	86	50.6%
6+	42	24.7%
Number of normal deliveries		
None	89	52.4%
1–2	41	24.1%
3–4	29	17.1%
5+	11	6.5%
Number of CS		
1	66	38.8%
23	84	49.4%
4–6	20	11.8%
Number of children		
1–2	63	37.1%
3–4	65	38.2%
5+	42	24.7%
Medical and drug history		
History of contraceptives use		
Oral contraceptive	61	35.9%
Hormonal therapy †	18	10.6%
None of them	91	53.5%
History of orthopedic trauma		
No	138	81.2%
Yes	24	14.1%
Do not remember	8	4.7%
History of pregnancy-induced hypertension		
No	129	75.9%
Yes	41	24.1%
Labor induction exceeded 24 hours		
No	131	77.1%
Yes	30	17.6%
Do not remember	9	5.3%
Physical activity during 24 hours after labor		
No	10	5.9%
Yes	160	94.1%
Medications during pregnancy		
Folic acid	169	99.4%
Iron	165	97.1%
Ca	109	64.1%
Vitamin D	47	27.6%
Aspirin	8	4.7%
Vitamin B12	4	2.4%
Omega 3	12	7.1%
Others	8	4.7%

†Any drug formula containing estrogen.

**Table 2:** Causes of suboptimal adherence to LMWH†.

Causes of suboptimal adherence	No	%
Perceived lack of necessity	16	44.4%
Forgetting	11	30.6%
A load of going to the healthcare institution	10	27.8%
Others	9	25%
Fear of needles	4	11.1%

†LMWH: enoxaparin.

**Table 3:** The distribution of parturients' adherence to LMWH postdischarge after cesarean delivery by their demographic and clinical data.

Demographic and clinical data	Total		Adherence to LMWH postdischarge				*P* value
			Fully adherent		Suboptimal adherent		
	No	%	No	%	No	%	
Age in years							.910
<30	52	30.6%	40	29.9%	12	33.3%	
30–39	90	52.9%	72	53.7%	18	50%	
40+	28	16.5%	22	16.4%	6	16.7%	
Educational level							.557
Below secondary	33	19.4%	27	20.1%	6	16.7%	
Secondary	67	39.4%	50	37.3%	17	47.2%	
University	70	41.2%	57	42.6%	13	36.1%	
Monthly income							.728
<10000 SR	122	71.8%	97	72.4%	25	69.4%	
>10000 SR	48	28.2%	37	27.6%	11	30.6%	
Body mass index							.777
Normal weight	49	28.8%	39	29.1%	10	27.8%	
Overweight	49	28.8%	40	29.9%	9	25%	
Obese	72	42.4%	55	41%	17	47.2%	
Comorbidities							.509†
None	112	65.9%	91	62.6%	21	56.8%	
DM	10	5.9%	8	5.4%	2	5.4%	
HTN	19	11.2%	12	8.2%	7	18.9%	
Anemia	27	15.9%	22	15.1%	5	13.5%	
Hypothyroidism	4	2.4%	3	4.3%	1	2.7%	
Others	10	5.9%	9	6.2%	1	2.7%	

*P:* Pearson X^2^ test. †: Exact probability test, ^∗^*P* < 0.05 (significant).

**Table 4:** Distribution of parturients' adherence to LMWH postdischarge by their gynecological and obstetric data.

O&G data	Total		Adherence to LMWH postdischarge				*P* value
			Fully adherent		Suboptimal adherent		
	No	%	No	%	No	%	
Gravidity							.924
1–2	42	24.7%	34	25.4%	8	22.2%	
3–5	86	50.6%	67	50%	19	52.8%	
6+	42	24.7%	33	24.6%	9	25%	
Number of normal deliveries							.215
None	89	52.4%	68	50.7%	21	58.3%	
1–2	41	24.1%	37	27.7%	4	11.1%	
3–4	29	17.1%	21	15.7%	8	22.2%	
5+	11	6.5%	8	5.9%	3	8.3%	
Number of C.Ss							.735
1 time	66	38.8%	50	37.3%	16	44.45%	
2–3	84	49.4%	68	50.7%	16	44.45%	
4–6	20	11.8%	16	12%	4	11.1%	
Number of children							.439
1–2	63	37.1%	51	38.1%	12	33.3%	
3–4	65	38.2%	48	35.8%	17	47.3%	
5+	42	24.7%	35	26.1%	7	19.4%	

*P:* Pearson X^2^ test.

**Table 5:** Distribution of parturients' adherence to LMWH postdischarge by their experiences and views regarding LMWH.

Experiences and views regarding LMWH			Adherence to LMWH postdischarge				*P* value
	Total		Fully-adherent		Suboptimal adherent		
	No	%	No	%	No	%	
The causes and method of drug intake was explained							.967
No	40	23.5%	31	23.1%	9	25%	
By pharmacist	9	5.3%	7	5.2%	2	5.6%	
By physician	121	71.2%	96	71.7%	25	69.4%	
First time to use LMWH							.340
No	33	19.4%	24	17.9%	9	25%	
Yes	137	80.6%	110	82.1%	27	75%	
If yes, frequency of previously receiving LMWH							.049∗
One	19	54.5%	15	11.1%	4	11.1%	
Two	10	30.3%	5	3.7%	5	13.9%	
Three	4	12.1%	4	3%	0	0.0%	
Had side effects due to the given drug							.381
No	153	90.0%	122	91%	31	86%	
Yes	17	10.0%	12	9%	5	14%	
Who does give you the injection?							.001∗†
Did not have the injection	7	4.1%	0	0.0%	7	19.4%	
My self	51	30.0%	45	33.6%	6	16.7%	
Family member	57	33.5%	47	35%	10	27.8%	
Health care staff	55	32.4%	42	31.4%	13	36.1%	

*P*: Pearson X^2^ test. †: Exact probability test.

**Table 6:** Distribution of parturients' adherence to LMWH postdischarge by their prescribed and taken doses.

Doses	Adherence to thromboprophylaxis after cesarean delivery				Total		*P* value
	Adherent		Nonadherent				
	Mean	SD	Mean	SD	Mean	SD	
Number of doses prescribed	7.62	1.09	7.75	1.83	7.65	1.28	.851
Number of doses actually taken	7.36	1.60	3.86	2.65	6.62	2.35	.001^∗^

*P*: Independent samples *t*-test. ^∗^*P* < 0.05 (significant).

## Data Availability

The data used to support the findings of this study are included within the article.

## Additional Points

*What is known*. The cesarean section increases the risk of DVT in some patients, therefore; those patients are given postcesarean LMWH thromboprophylaxis. The adherence rate to LMWH after cesarean section is varied in different published studies. Some studies showed a high adherence rate while others reported a low adherence rate. *What is new*. To the best of our knowledge, no study was conducted in Saudi Arabia to assess women's adherence and their experiences with LMWH thromboprophylaxis after discharge from the hospital. Therefore, we conducted this study to assess postcesarean parturients' adherence to the LMWH thromboprophylaxis regimen. We investigated the causes that influence adherence to the LMWH thromboprophylaxis regime. Also, the results of this study may give the health care authorities an idea about the current situation and how it could be improved and potentially decrease the risk of DVT in those patients.
